The article "Analysis of Music Retrieval Based on Emotional Tags Environment" was retracted in 2023. Reasons: unreliable results or conclusions; concerns about the data; concerns about the results or conclusions; concerns about the peer review.

# Analysis of Music Retrieval Based on Emotional Tags Environment

**DOI:** 10.1155/2022/4670963

**Published:** 2022-08-16

**Authors:** Nuan Bao

**Affiliations:** ^1^Institute of Music, Theater and Choreography, The Herzen State Pedagogical University, Saint Petersburg 191186, Russia; ^2^Xuzhou Kindergarten Teachers College, Xuzhou 221004, China

## Abstract

In general, tags are used to interpret the content of music, while the music itself expresses emotion. The emotional information conveyed by the same music is described by a large number of emotion tags in various ways. This paper proposes and establishes an algorithm for music retrieval based on emotional tags. By modelling user emotional tags and music, a bipartite graph with emotional tags and music as nodes is first created. The tags and semantic similarity between the music are then calculated using the T_SimRank algorithm, and the popularity of the music is calculated using the T_PageRank algorithm. Finally, the two methods are combined using the concept of ranking learning to produce the final ranking of the music. Experiments demonstrate that the method suggested in this paper can better satisfy user retrieval needs than conventional cosine similarity and tag co-occurrence-based similarity methods and that the fusion of multiple methods is preferable to a single method.

## 1. Introduction

Music has always been a necessary and significant part of people's lives as a means of expressing inner emotions. As Internet technology advances, more people are turning to the Web to pass their free time by watching movies, listening to music, and reading electronic novels. The Internet has developed into a significant medium for the distribution of musical materials. A keyword-based approach is essentially all that is required to retrieve qualified music works from the music library. Traditional music retrieval is primarily based on the external characteristics of music, such as title, songwriter, singer, lyrics keywords, and so on. Users who use text search must keep in mind the pertinent information in order to be able to retrieve music. The traditional music retrieval method cannot satisfy a user's needs when he hears a good song in a mall or on the highway because he is unable to identify the singer, the song's title, or other relevant information. In the creation of music, emotions are crucial. People express their inner emotions through music, making emotional analysis of music a significant area of study for psychologists and musicologists.

Reference [1] investigated the relationship between people's understanding, mood, and music genes. The objective is to create a model of gene-maturity-environment interaction in the context of musical ability as a way to understand how tendencies, brain development, and experience interact. To achieve the unity of music features and advertising features, reference [2] investigates the relationship between the emotional characteristics of music and advertising effects; reference [3] suggests a method of music therapy for the emotional needs of the elderly. Reference [4] investigated how to convey individualised emotional traits through music instruction; Chowdhury et al. [5] employed machine learning algorithms to foretell the emotional elements of musical compositions; and Hong and Luo [6] studied the ways that musical emotional characteristics are taught and talked about some typical ways that these musical characteristics are taught.

Many academics conduct extensive research in the area of music emotion labelling. For instance, Liu et al. [7] and Chaudhary et al. [8] proposed using a recurrent neural network to identify music emotion. References [9, 10] investigated the issue of music emotion classification and came to a more accurate conclusion by classifying music emotion from lyrics and audio using corpus-based, literature through audio and audiovisual methods. Label retrieval can be used in a variety of information search fields, including feature fusion and font retrieval (see reference [11]). Won et al. [12] created label-based music retrieval by incorporating cross-modal retrieval tasks, in order to enhance the inspection's outcomes. It increases the accuracy and effectiveness of music library browsing.

The ranking of query results is an important research topic in various search engines because it is directly related to the needs of the query personnel for the query system. For instance, reference [13] investigated the ranking of news recommendation results; reference [14] investigated the impact of semantic similarity on retrieval outcomes; and reference [13] discovered that “popularity” is a crucial indicator that influences the outcomes of music retrieval. References [15, 16] investigated the factors influencing music popularity and created models that corresponded to their findings. Reference [17] uses supervised deep learning to implement the retrieval of music videos, and [18] used vector machines to categorise and process the music retrieval results.

This study builds a bipartite graph with emotional tags and music as nodes, applies the T_SimRank algorithm to determine the semantic similarity between tags and music, and then applies the calculation of semantic similarity of short texts to determine the semantic similarity between search tag strings and music. The other function, popularity, returns the song's “popularity.” The popularity of music is incorporated into music retrieval, which significantly boosts the effectiveness of music retrieval. This paper develops the T SimRan algorithm and obtains the T_PageRank algorithm for music popularity ranking while taking into account the tag's own popularity data. The final ranking of music is determined by combining the two factors of similarity and popularity, and ranking learning is used to determine this ranking in order to improve user experience.

## 2. Semantic Similarity Calculation of Tags

These tags represent the user's perception and analysis of the music. The article's emotional tags also include words such as “love,” “family,” and others that can convey emotional information, in addition to emotional words with conventional meanings such as “sad” and “happy.” The same song has several different emotional tags. For instance, “Simple Love” by Jay Chou contains a range of feelings, including “beautiful,” “leisure,” “first love,” “summer,” “quiet,” “happy,” “tenderness,” and so on. The same emotional tag can be used to describe several songs at once; for example, “Sad” can be used to describe several songs by Liang Jingru, including “Pain That Can Breathe,” “Unfortunately Not You,” “It's Always Quiet,” and others. There is a “many-to-many” relationship between tags and music. Labels and songs are represented as nodes in the bipartite graph in Figure 1, and the edges represent the labelling relationships between them.

In Figure 1, the tags “sad” and “sad” are marked with three pieces of music: “Got a little hurt – Asan,” “After I leave – Jane Zhang,” and “Li Song – Xin Orchestra,” then, which of these two tags, there is a certain semantic relationship between them. Similarly, if the music “Got a little hurt – ASan” and “After I leave – Jane Zhang” are marked as “sad” and “feel sorry” at the same time, then there is also a relationship between the two pieces of music—a certain degree of similarity. Music retrieval is based on tag semantic similarity can retrieve music that does not contain the tag but has a high degree of similarity to it. For example, when searching with the tag “feel sorry,” although the music “breathing pain – Liang Jingru” is not marked as “feel sorry,” all its tags are very similar to “feel sorry.” Higher similarity is ranked ahead of other music marked as “feel sorry.”

### 2.1. Semantic Similarity Based on Tag Cooccurrence

Each piece of music contains a certain number of tags. These tags reflect the emotion, theme, style, and other information of the music from different angles. Semantic similarity based on tag co-occurrence refers to the semantic similarity of tags obtained by calculating the co-occurrence frequency of tags. Reference [13] used this method to calculate the semantic similarity of tags. The formula is as follows:

(1) $$\begin{array}{c} \text{Co}\_\text{Sim}\left(t_{i},t_{j}\right)=\frac{\left|t_{i}\cap t_{j}\right|}{\left|t_{i}\cup t_{j}\right|}, \end{array}$$

where |*t*_*i*_∩*t*_*j*_| represents the number of music labeled *t*_*i*_ and *t*_*j*_ at the same time and |*t*_*i*_ ∪ *t*_*j*_| represents the number of music labeled *t*_*i*_ or *t*_*j*_.

### 2.2. Semantic Similarity Based on T_SimRank Algorithm

Jeh and Widom proposed the SimRank algorithm in 2002, which uses the global information of the graph to calculate any two nodes. The idea of SimRank is the neighbour nodes of two nodes are similar, so the two nodes are also similar.

According to its idea, this paper proposes the T_SimRank algorithm. The basic ideas are as follows:

1. Assuming that the two labels are similar, then the music they respectively label is also similar
2. Assuming that two pieces of music are similar, then the tags they have are also similar
3. Any tag has the greatest similarity with itself
4. Any piece of music has the greatest similarity to itself

Iterative processes are used in T_SimRank. The basic operation of the T_SimRank algorithm is shown in Table 1, where N_tag_ stands for the number of tags, N_music_ for the number of songs, S_tag_ for the similarity matrix of tags, and Stag(*t*_*i*_, *t*_*j*_) for the tag. *t*_*i*_ and *t*_*j*_ share a semantic similarity. Music's similarity matrix is denoted by Smusic, and the semantic similarity between musics si and sj is denoted by Smusic represents the likelihood of a transition from label ti to music sj, and Pt->*s* (*s*) is the transition probability matrix of order N_tag_ × N_music_, P_t->s_(*t*_*i*_, *s*_*j*_) denotes the probability of a transition from si to tj, and Ps->*t* is the transition probability matrix of order N_music_ × N_tag_, P_t->s_(*s*_*j*_, *t*_*i*_).

Assuming convergence is achieved after *k* iterations, the time complexity of T_SimRank is *O*(*N*_*tag*_^2^*∗N*_*music*_^2^*∗k*). Taking Figure 1 as an example, both c1 and c2 are set to 1. After the first iteration, the similarity between labels is shown in Figure 2.

In tag-based retrieval, tags are used as search terms for querying. In the paper, *q*={*q*_1_, *q*_2_, *q*_3_,…, *q*_*n*_} is used to represent the query string *q*, and *T*(*s*)={*t*_1_, *t*_2_, *t*_3_,…, *t*_*m*_} is used to represent the label set of music *s*, and then, the similarity between *q* and *s* is

(2) $$\begin{array}{c} \text{sim}\left(q,s\right)=\sum_{i=1}^{n}\sum_{T\in S}S_{\text{tag}}\left(q_{i},t\right). \end{array}$$

In this paper, considering the contribution of tags to music, the short text semantic similarity calculation method in Reference [14] introduces the idf value into the following formula:

(3) $$\begin{array}{c} \text{sim}\left(q,s\right)=\frac{1}{2}\left(\frac{\sum_{i=1}^{n}\max S_{\text{tag}}\left(q_{i},s\right)\times \text{idf}\left(q_{i}\right)}{\sum_{i=1}^{N}\text{idf}\left(q_{i}\right)}+\frac{\sum_{j=1}^{m}\max S_{\text{tag}}\left(t_{j},q\right)\times \text{idf}\left(t_{j}\right)}{\sum_{j=1}^{m}\text{idf}\left(t_{j}\right)}\right). \end{array}$$

## 3. Music Popularity Based on T_PageRank

### 3.1. PageRank Algorithm

Sergey Brin and Lawrence Page, the co-founders of Google, proposed the PageRank algorithm in 1998. It is a formula used to determine page rankings. The random walk principle serves as the foundation of its algorithm. An example of an irregular variation is a random walk. Every step in this process of change is completely random, just like when someone is out drinking. Applying the random walk process to a graph entails starting at any node and moving randomly to each of its neighbouring points. It is possible to repeat this random process. The percentage of time the person spends at each node will stabilise if the graph is irreducible and aperiodic.

The fundamental tenet of PageRank is that significant vertices must be frequently visited if a random walk in a network is to be taken into account. By calculating the access probability of each vertex, it is possible to determine the significance of each vertex. Pages linked from numerous high-quality pages are assumed to be high-quality pages by the PageRank algorithm. Its traits are linked to the link structure between web pages rather than the user's query process. It is clear from the assumptions based on the PageRank algorithm that a web page's PR value depends on three variables: the quantity of links pointing to the page, the quantity of links pointing to the page, and the quality (importance) of the page linked to.

The PageRank algorithm is frequently translated into an iterative calculation process that involves multiplying two two-dimensional matrices. The initial weights of all nodes are typically assumed to be the same. Each web page's first iteration ranking is then determined based on this initial weight and the direct conversion probability matrix of all nodes, and the second ranking is determined in accordance with the first iteration ranking.

The PageRank algorithm is an iterative procedure that mimics users' web page browsing behaviour. The user is assumed to begin on one web page, choose at random one of its linked web pages to browse, and then repeat the process. When enough time has passed, the longer a user spends on a particular web page, the more likely it is that the PR value will tend to converge.

Page theoretically proves that no matter how the initial value is selected, the PageRank algorithm can guarantee that the estimated values of all page rankings can converge to their true values. The random walk idea used by the PageRank algorithm is widely used in various research fields, such as the motion law of molecules in physics, the simulation of animal foraging paths in ecology, and the fluctuation law of stocks in economics. In the field, random walk models can be used in social networks, recommender systems, personalised retrieval, classification, clustering, and automatic summarisation.

### 3.2. T_PageRank Algorithm

Reference [19] uses the PageRank principle, uses the tag co-occurrence relationship between music as the link between the music to obtain the music popularity based on tags, and adds the music popularity to the retrieval, which improves the retrieval accuracy. However, it does not take into account the influence of the popularity of the tag itself on music, that is, when users are listening to music, it is easier to choose to link to new music from a more popular tag. In this paper, the hotness information of tags is added to the algorithm of literature, and the T_PageRank algorithm is obtained, which is based on the following two assumptions:

1. The stronger a piece of music is linked to other music, the higher the popularity of the music
2. The higher the popularity of the music link, the higher the popularity of the music

In the above description, the link degree of music mainly includes the number of co-occurring tags and the popularity of tags. The popularity of a label usually refers to the number of times a label is marked. In this paper, it is represented by the number of music marked by a label, that is, the more music a label is marked, the higher the popularity of the label. Hot(*t*_*i*_) represents the hotness of the tag *t*_*i*_, and N(*t*_*i*_) represents the number of music marked by the tag. That is, Hot(*t*_*i*_) = N(*t*_*i*_). Construct a graph G<V, E>, where V represents the set of nodes, that is, the set of music. E represents the degree of music link based on tags, which is obtained by the following formula:

(4) $$\begin{array}{c} w_{ij}=\frac{\sum_{m=1}^{\left|T_{i}\cap T_{j}\right|}\text{Hot}\left(t_{m}\right)}{\sum_{n=1}^{\left|T_{i}\cup T_{j}\right|}\text{Hot}\left(t_{n}\right)}, \end{array}$$

where w_*ij*_ represents the weight of the edge between nodes

*v*_*i*_ and *v*_*j*_ and *T*_*i*_ and *T*_*j*_ represent the label sets of *v*_*i*_  and *v*_*j*_, respectively. |*T*_*i*_∩*T*_*j*_| represents the number of intersections of tag sets *T*_*i*_ and *T*_*j*_, and |*T*_*i*_ ∪ *T*_*j*_| represents the number of unions of *T*_*i*_ and *T*_*j*_. Similar to PageRank, T_PageRank is also an iterative algorithm, and its core algorithm is shown in formula (5). After iteratively converges, Hot(*v*_*i*_) represents the final hotness of music *v*_*i*_. *d* is the damping coefficient, and its value is 0.83. In(*v*_*i*_) represents the set of nodes pointed to *v*_*i*_, and Out(*v*_*j*_) represents the set of nodes pointed to by *v*_*j*_; in this paper, In(*v*_*i*_)=Out(*v*_*j*_).

(5) $$\begin{array}{c} \text{Hot}{\left(v_{i}\right)}^{p+1}=\left(1-d\right)+d*\sum_{v_{j}\in \text{In}\left(v_{i}\right)}\text{Hot}{\left(v_{j}\right)}^{p}*\frac{w_{ij}}{\sum_{v_{k}\in \text{Out}\left(v_{j}\right)}W_{jk}}. \end{array}$$

Figure 3 is a subschematic diagram of graph G, which includes eight song nodes and the degree of mutual linking.

The iterative T_PageRank algorithm uses the graph structure. Assuming that convergence is attained after *k* iterations, *n* is the total number of music nodes, and d2 is used to represent the average number of adjacent points of music nodes. The algorithm's time complexity is O(knd2), and its space complexity is O(1). O is the complexity (n2). The initial weight of the node will influence the number of iterations, and the number of times the music is labeled can reflect the popularity of the music to some extent, even though the node weight after the convergence of the T_PageRank algorithm has nothing to do with the node's initial weight value. To cut down on the number of calculation iterations as much as possible, the number is used as the initial weight of each node.

## 4. Sentiment Tag Recommendations for New Music

### 4.1. New Music Recommendation Mode

The object of music retrieval research based on emotional tags is the emotional tag of music, which depends on the user's annotation and is a “dominant” gene displayed by a song under the premise of being followed by the user. However, for a new song Music, in the case that it is not yet familiar to the public, its emotional information is still contained in the music with a “hidden” feature. Therefore, how to use the lyrics, audio, and other information of the song to dig out new music is the subject of this paper to label some “virtual” emotional tags for a new piece of music so that it can be timely returned to the user in the music retrieval based on emotional tags.

In order to solve the problem of the lack of emotional tags for new music, this paper uses typical content-based tag recommendation technology.

First, find the list of songs with the most similar emotions by calculating the emotional similarity between the lyrics of the songs to be recommended and the known songs.

Then, according to the similarity ranking, the corresponding label is regarded as the “virtual” label of the song with the unknown label.

The new music of the tag can also participate in the tag-based music retrieval process.

The emotional tag prediction method of music can be transformed into a tag recommendation for new music. Tag recommendation technology is a new research field with the birth of WEB2.0. In social networks, user information is usually considered to do some personalised recommendation services. The commonly used methods include content-based recommendation, collaborative filtering-based recommendation, and graph structure-based recommendation.

The main idea of the collaborative filtering algorithm is to recommend for the same group with similar points of interest, which takes the user's evaluation of the item as the basis for interest evaluation, and similar users make corresponding interest in the item according to the evaluation of similar users. At present, most of the recommendation algorithms of common e-commerce platform shopping websites use collaborative filtering algorithms.

A content-based recommendation typically identifies known resources that are comparable to the resources to be recommended, calculates their similarities, and then suggests the label of the resource with the greatest similarity. Tess, a resource content-based tag recommendation system, was created by Oliveira et al. To recommend tags based on the word frequency ranking of tags in related documents, the cosine similarity calculation is first used to identify the document set that is most similar to the known document. Technology that uses content-based recommendations can more effectively address cold start and data sparsity issues, as well as perform tag recommendation for newly added resources or users who do not yet have tag records in the system.

The recommendation technology based on collaborative filtering mainly analyses user interests, finds similar (interested) users of the user to be recommended in the user group, and integrates the evaluations of these similar users on certain information to form the system's preference for the specified user. At present, some social networking sites such as Amazon, CDNow, YouTube, Flickr, and so on have adopted the technology of collaborative filtering to improve service quality. The label recommendation method of collaborative filtering relies on the historical data marked by users and can better recommend personalised labels by analysing the user interest model, but the quality of label recommendation depends on historical data, which easily leads to data sparsity and cold start problems.

### 4.2. New Music Recommendation Mode

The collaborative filtering algorithm, when compared to other recommendation algorithms, has several clear advantages: it is recommended based on the experiences of similar or similar users, saving time spent analyzing the qualities and attributes of the items, avoiding the need to evaluate and assess the content of the items, and increasing the effectiveness of grouping. In a short amount of time, accurate recommendations are finished. Its flaws are also clear at the same time. New users lack behavioural information and some experience values when making recommendations. It is simple to create some mandatory and irrational recommendations when splitting groups, which has poor recommendation effects for some people. The collaborative filtering algorithm requires a significant amount of historical data collection for a recommendation. The execution performance of the collaborative filtering algorithm will degrade after a large number of calculations and with the ongoing expansion of the item database.

There are a variety of algorithms for making recommendations, such as algorithms based on collaborative filtering, association rules, and content. The collaborative filtering algorithm is used by the music system under study in this system. These are the primary causes: based on content suggestions, the selection of music frequently depends on the same kind of learning of similar users, though it is typically realised through the user's retrieval records. Before appreciating a piece of music, one is only aware of its title, lyrics, and classification of related titles, among other things. It is necessary to take into account the learning experiences of other relevant personnel because, limited to personal knowledge, there is some variation in the music selection. As a result, even though the content-based recommendation is recommended from the user's retrieval behaviour, it has some advantages in online music recommendation. Although there is some overlap between the points, it is only to a certain extent due to the possibility of users selecting music. As a result, using correlation analysis alone to suggest music can lead to some unintended consequences.

### 4.3. New Music Recommendation Mode

Throughout the process, it is used as the training set. Through the SVM classifier, the song to be recommended finds its emotional category, finds the song with the highest similarity to itself in the emotional category, and uses its label as the candidate.

Select the Recommended tab. The whole tag recommendation process is as follows:

1. Use the IR emotion ontology library to obtain the emotion vector of the lyrics
2. Use the SVM classifier to train a multisentiment classification model
3. Input the emotion space vector of the song to be recommended and use the SVM classifier to predict the emotion to which the song belongs the main category of sense
4. Use the cosine similarity formula to calculate the emotional space vector of the song to be recommended and all the songs of the main category similarity
5. Sort the similarity and take the top M songs with the highest similarity as the similar songs
6. Calculate the tags of similar songs according to the similarity weight and select the top M as candidate tags to recommend to songs

## 5. Experiment and Results

### 5.1. Experimental Data Set

This paper obtains 35,365 pieces of music from “Google Music” and all the labels in the “Music Emotion” category as the experimental corpus. At the same time, 20 groups of tag query strings are set, of which 10 groups are positive emotions and the other 10 groups are negative emotions, and the number of tags in each group of query strings varies from 1 to 5 tags. In the form of a questionnaire, 10 respondents were asked to recommend the 100 pieces of music they thought they were most satisfied with and then set the music to 1–5 relevant levels according to the number of recommendations, where 1 means irrelevant, that is, the number of recommendations is 0–2 that indicates weak correlation, and the number of recommendations is less than or equal to 2; 3 means partial correlation, and the number of recommendations is 3–5 times; 4 means relatively relevant, and the number of recommendations is 6–8 times; and 5 means very relevant, and the number of recommendations is 9–10 times. Considering the influence of the relevance of music and the location of the returned results on the user experience, this paper chooses to use the NDCG@N value as the evaluation index.

### 5.2. Experimental Design

This paper uses the Ranking SVM [20] ranking model to train the weights of each feature, and all parameters including the loss function use default values. A total of three sets of comparative experiments are designed in this paper as follows:

1. Comparison of cosine (consin) similarity, tag co-occurrence (Co_Tags) similarity, and T_SimRank results. Among them, the consin similarity is to construct a vector space model by considering the tag string as a short text and each tag as a feature item and sort by calculating the cosine similarity between the query tag string and the music tag string.
2. The three similarity calculation methods are added with T_PageRank heat information (represented by consin^*∗*^, Co_Tags^*∗*^, and T_SimRank^*∗*^, respectively, in the paper) for comparison. In the experiment, 6 groups of positive emotions and 6 groups of negative emotions are selected, a total of 12 groups of query results. As the training set, the remaining 8 groups are used as the test set.
3. consin versus consin^*∗*^
4. co_Tags versus Co_Tags^*∗*^
5. TSimRank versus TSimRank^*∗*^
6. consin^*∗*^, Co_Tags^*∗*^, r_SimRank^*∗*^ comparison.
7. For experiments (i) and (ii), although the average NDCG value of T_SimRank is higher than the similarity of consin and Co_Tags, it is not as effective as the latter for the query string “natural, fresh, and enjoyable.” When T SimRank calculates the similarity, it will have an advantage for songs with a relatively small number of tags. However, the number of tags is not only for some new songs but also for some songs that are very unpopular. Therefore, this paper uses sorting learning to compare the previous three methods by combining two or all three, hoping to achieve better results.

### 5.3. Analysis of Results

Figures 4 and 5 are the average NDCG values of experiments (i) and (ii), respectively. Through analysis, it can be seen that the effect of T_SimRank is significantly better than that of consin similarity and Co_Tags similarity. After adding T_PageRank heat information, the three methods results were improved, with T_SimRank^*∗*^ performing the best.

For each method in Figure 4, the paper analyses the return result of each query string; the results of 18 query strings are in line with the curve trend in Figure 4, but in the results returned by the query strings “natural, fresh, enjoyment” and “beautiful, relaxing, mind, life,” T_SimRank is not as good as consin similarity and Co_Tags similarity. After analysis, it is found that the returned results of these two query strings contain some relatively unpopular songs. This is because TSimRank considers the average similarity of all songs related to the two tags when calculating the similarity. In this method, there are certain advantages for some songs with a relatively small number of tags. In Figure 5, the paper selects 6 groups of positive emotions and 6 groups of negative emotions, a total of 12 groups of query results as the training set, and the remaining 8 groups are used as the test set. By comparison, it is found that the effect of pairwise fusion is significantly better than the return result of a single method, and the fusion effect of the three is the best.

## 6. Conclusions

Since music is an expression of emotion, users can find songs that suit their mood by describing them using music retrieval based on emotion tags. By determining the semantic similarity between tags and the popularity of music, the T_SimRank algorithm and T_PageRank algorithm proposed in this paper can better serve the user's retrieval needs than the conventional cosine similarity and the similarity method based on tag co-occurrence. The ranking learning approach combines several approaches, and the result is superior to using just one. In order to improve the effectiveness of music retrieval, we will think about incorporating the emotional information conveyed by a song's melody, genre, and other information into the algorithm suggested in this paper.

## Figures and Tables

**Figure 1:** Diagram of the relationship between labels and music.

**Figure 2:** Similarity between labels after the first iteration.

**Figure 3:** Schematic representation of subgraphs of graph G.

**Figure 4:** Average NDCG of a single method.

**Figure 5:** Average NDCG values fused by multiple methods.

**Table 1:** T_SimRank algorithm.

Algorithm: T_SimRank

Input: N_tag_, N_music_, P_t->s_, P_s->t,_ convergence threshold *c*_*1*_ and *c*_*2*_

Step1: Initialisation: $S_{\text{tag}}\left(t_{i,}t_{j}\right)=\left\{\begin{array}{cc} 1, & i=j,\\ 0, & i\neq j, \end{array}\right)$$S_{\text{music}}\left(S_{i},S_{j}\right)=\left\{\begin{array}{cc} 1, & i=j,\\ 0, & i\neq j. \end{array}\right)$
Step2: Do{*S*_tag_^*k*+1^(*t*_*i*_, *t*_*j*_)=*c*_1_∑_*m*=1_^|*N*_music_|^∑_*n*=1_^|*N*_music_|^*P*_*t*⟶*s*_(*t*_*i*_, *S*_*m*_)*S*_music_^*k*^(*S*_*m*_, *S*_*n*_), *S*_music_^*k*+1^(*S*_*i*_, *S*_*j*_)=*c*_2_∑_*m*=1_^|*N*_tag_|^∑_*n*=1_^|*N*_tag_|^*P*_*s*⟶*t*_(*S*_*i*_, *t*_*m*_)*P*_*s*⟶*t*_(*S*_*j*_, *S*_*n*_)*S*_tag_^*k*^(*t*_*m*_, *t*_*n*_)} until (*S*_tag_^*k*^(*t*_*i*_, *t*_*j*_) − *S*_tag_^*k*−1^(*t*_*i*_, *t*_*j*_) ≤ *ɛ*_1_&&|*S*_music_^*k*^(*S*_*i*_, *S*_*j*_) − *S*_music_^*k*−1^(*S*_*i*_, *S*_*j*_)| ≤ *ɛ*_2_).

Output: Label similarity matrix S_tag_, music similarity matrix S_music_

## Data Availability

The data used to support the findings of this study are available from the author upon request.

## References

[1] Penhune V. B. (2020). A gene-maturation-environment model for understanding sensitive period effects in musical training. *Current opinion in behavioral sciences*.

[2] Hou J., Zhao X., Zheng J. (2019). The impact of consistency between the emotional feature of advertising music and brand personality on brand experience. *Journal of Management Analytics*.

[3] Jang S., Kunde L. (2021). A systematic review of music therapy interventions used to address emotional needs of older adults. *The Arts in Psychotherapy*.

[4] Bonastre C., Timmers R. (2021). Comparison of beliefs about teaching and learning of emotional expression in music performance between Spanish and English HE students of music. *Psychology of Music*.

[5] Chowdhury S., Vall A., Haunschmid V., Widmer G. (2019). Towards explainable music emotion recognition: the route via mid-level features. https://arxiv.org/abs/1907.03572.

[6] Hong H., Luo W. (2021). *The Method of Emotional Education in Music Teaching*.

[7] Liu H., Fang Y., Huang Q. Music emotion recognition using a variant of recurrent neural network.

[8] Chaudhary D., Singh N. P., Singh S. (2021). Development of music emotion classification system using convolution neural network. *International Journal of Speech Technology*.

[9] Rachman F. H., Sarno R., Fatichah C. (2018). Music emotion classification based on lyrics-audio using corpus based emotion. *International Journal of Electrical and Computer Engineering*.

[10] Kostiuk B., Costa Y. M. G., Britto A., Hu X., Silla C. Multi-label emotion classification in music videos using ensembles of audio and video features.

[11] Chen T., Wang Z., Xu N., Jin H., Luo J. Large-scale tag-based font retrieval with generative feature learning.

[12] Won M., Oramas S., Nieto O., Gouyon F., Serra X. Multimodal metric learning for tag-based music retrieval.

[13] Li J., Lin H., Zhou L. (2010). Emotion tag based music retrieval algorithm. *Asia Information Retrieval Symposium*.

[14] Nguyen H. T., Duong P. H., Cambria E. (2019). Learning short-text semantic similarity with word embeddings and external knowledge sources. *Knowledge-Based Systems*.

[15] Lee J., Lee J. S. (2018). Music popularity: metrics, characteristics, and audio-based prediction. *IEEE Transactions on Multimedia*.

[16] Araujo C., Soares V., de Cristo M. A. P., Giusti R. Predicting music popularity using music charts.

[17] Zeng D., Yi Yu, Oyama K. Audio-visual embedding for cross-modal music video retrieval through supervised deep CCA.

[18] Zhang B. O., Lin J. An efficient content based music retrieval algorithm.

[19] Klicpera J., Bojchevski A., Günnemann S. (2018). Predict then propagate: graph neural networks meet personalized pagerank. https://arxiv.org/abs/1810.05997.

[20] Chauhan V. K., Dahiya K., Sharma A. (2019). Problem formulations and solvers in linear SVM: a review. *Artificial Intelligence Review*.

